# A Media and Clinic Intervention to Increase Colorectal Cancer Screening in Ohio Appalachia

**DOI:** 10.1155/2015/943152

**Published:** 2015-10-05

**Authors:** Jessica L. Krok-Schoen, Mira L. Katz, Jill M. Oliveri, Gregory S. Young, Michael L. Pennell, Paul L. Reiter, Jesse J. Plascak, Michael D. Slater, Janice L. Krieger, Cathy M. Tatum, Electra D. Paskett

**Affiliations:** ^1^Comprehensive Cancer Center, The Ohio State University, 1590 N. High Street, Suite 525, Columbus, OH 43201, USA; ^2^Division of Cancer Prevention and Control, Department of Internal Medicine, College of Medicine, The Ohio State University, 395 W. 12th Avenue, Columbus, OH 43210, USA; ^3^Division of Health Behavior and Health Promotion, College of Public Health, The Ohio State University, 1841 Neil Avenue, Columbus, OH 43210, USA; ^4^Center for Biostatistics, The Ohio State University, 1800 Cannon Drive, Columbus, OH 43210, USA; ^5^Division of Biostatistics, College of Public Health, The Ohio State University, 1841 Neil Avenue, Columbus, OH 43210, USA; ^6^Biobehavioral Cancer Prevention and Control Training Program, University of Washington, P.O. Box 359455, Seattle, WA 98195, USA; ^7^School of Communication, The Ohio State University, 3022 Derby Hall, 154 N. Oval Mall, Columbus, OH 43210, USA; ^8^STEM Translational Communication Program, University of Florida, 2088 Weimer Hall, 1885 Stadium Road, Gainesville, FL 32611, USA; ^9^Division of Epidemiology, College of Public Health, The Ohio State University, 1841 Neil Avenue, Columbus, OH 43210, USA

## Abstract

*Objective*. To test the effectiveness of a colorectal cancer (CRC) screening intervention among adults living in Ohio Appalachia. *Methods*. We conducted a group-randomized trial of a county-level intervention among adults living in 12 Ohio Appalachian counties who received a media campaign and clinic intervention focused on either CRC screening or fruits and vegetables. Participants' percentage within CRC screening guidelines was assessed with cross-sectional surveys conducted annually for four years, and validated with medical record review of screening. *Results*. On average, screening data were obtained on 564 intervention and 559 comparison participants per year. There was no difference in the Wave 4 CRC screening rates of intervention and comparison counties (35.2% versus 31.4%). Multivariate analyses found that high perceived risk of CRC, willingness to have a CRC test if recommended by a doctor, doctor recommendation of a CRC screening test, and patient-physician communication about changes in bowel habits, family history of CRC, and eating fruits and vegetables were significant (*p* < 0.05) predictors of being within CRC screening guidelines. *Conclusions*. The intervention was not effective in increasing CRC rates among Ohio Appalachian adults. Future research should determine how media and clinic-based interventions can be modified to improve CRC screening rates among this underserved population.

## 1. Introduction

Colorectal cancer (CRC) is the third leading type of cancer and the second leading cause of cancer death among men and women in the United States [1]. Significant disparities in incidence, mortality, and survival rates exist among underserved populations for this disease [1–6]. Moreover, CRC screening modalities are less likely to be used regularly among underserved populations [4–6]. One underserved population that bears an excess burden of CRC is residents of Ohio Appalachia, a 32-county region in southern and eastern Ohio [6]. Rates of CRC incidence and mortality are approximately 17% and 18% higher, respectively, among Ohio Appalachian residents compared to the average age-adjusted US population in 2005 [7, 8]. Many factors common among residents living in Ohio Appalachia may contribute to CRC disparities, particularly limited access to cancer screening, low socioeconomic status (SES), and behavioral factors (poor diet, increased tobacco use) [2, 7, 9].

Screening and early detection have the potential to significantly reduce CRC incidence and mortality [10]. Previous media campaigns about CRC screening have resulted in greater reported exposure to messages about CRC screening [11, 12], increased intention to speak to doctors about CRC screening [12], and increased CRC screening [13, 14] at a relatively low cost per person screened [14]. The goal of this study was to implement and evaluate a county-level intervention consisting of media and clinic-level components to increase CRC screening in Ohio Appalachian residents.

## 2. Materials and Methods

This study used a group-randomized trial design. A CONSORT diagram (Figure 1) outlines the study design. Twelve Ohio Appalachian counties were stratified into three groups (high, medium, and low) based on the average percent of late stage CRC diagnoses (obtained from the Ohio Cancer Information Surveillance System). Within each of the groups, the four counties were randomized to either the intervention or comparison condition. Details regarding the development and design of the CRC screening intervention have been previously reported [15, 16]; however, we briefly describe the intervention components below.

### 2.1. Study Design

The effect of the intervention program, “Get Behind Your Health! Talk to Your Doctor About Colon Cancer Screening,” on CRC screening rates was evaluated, using telephone surveys of randomly selected residents in each of the 12 counties. Surveys were conducted annually for four years over a four-month period each year (preintervention (Wave 1), postmedia only (Wave 2), postclinic intervention only (Wave 3), and postcombination media and clinic intervention (Wave 4)), with medical record review (MRR) for those who reported completing a CRC screening test to validate self-reports of CRC screening behavior (fecal occult blood test (FOBT), flexible sigmoidoscopy, or colonoscopy).

The study was powered for a mixed model ANCOVA analysis [17] based on a comparison of Wave 4 screening rates. It was estimated that a sample size of 90 participants per county was needed to achieve 80% power to detect a difference of 10% in screening rates assuming a screening rate of 32% in the comparison arm (based on Ohio BRFSS data) and an Intraclass Correlation Coefficient (ICC) of 0.0046. Based on this calculation, 6 counties were randomized to each condition (intervention and comparison) and 90 residents from each county were recruited for each survey.

### 2.2. Eligibility and Recruitment

The following methodology was used for each wave of data collection. Names of residents in each of the 12 Ohio Appalachian counties were randomly selected from InfoUSA County Directories. Names were sampled with replacement at each wave. Potentially eligible participants were mailed a study packet that included a recruitment letter and a study information handout outlining key elements of standard informed consent and HIPAA authorization documents. Five days after the letters were sent, trained interviewers called potential participants and described the study, addressed concerns, answered questions, and assessed eligibility. Verbal informed consent and HIPAA authorization were obtained, and then the cross-sectional survey was administered.

Participants were eligible if they (1) were men and women aged 51–75 years; (2) had a working phone number; (3) were English-speaking and able to give informed consent; (4) were a resident of one of the 12 Ohio Appalachian counties at the time of the interview; (5) had no prior history of invasive cancer (including CRC), polyps, inflammatory bowel disease, Crohn's disease, or colitis; and (6) had no strong family history of polyps, CRC, or hereditary CRC syndromes. Participants received a $10 gift card after completing each survey as an expression of appreciation for their time. A medical record release form was also sent to each participant with a postage-paid envelope to return the completed form to the study office. Informed consent procedures and the study protocol were approved by the Institutional Review Board of The Ohio State University.

### 2.3. Intervention

The “Get Behind Your Health! Talk to Your Doctor About Colon Cancer Screening” intervention utilized a community-based participatory research approach to develop and pilot the CRC screening intervention. Based on results from a community assessment and in partnership with community members from Ohio Appalachia, a culturally sensitive media campaign that focused on increasing CRC screening was developed for use in the current study [15].

The intervention consisted of two main components: (1) a media campaign and (2) a clinic intervention [15, 16]. The intervention was based on health behavior theories, including the Health Belief Model (HBM) [18], the Theory of Reasoned Action (TRA) [19], Social Cognitive Theory (SCT) [20, 21], and Attitude Accessibility Theory (AAT) [22]. The theoretical constructs included in the campaign were as follows: HBM, which helped identify perceived benefits and barriers associated with CRC screening; TRA, which helped identify specific beliefs that must be reinforced or countered (e.g., community members talk about media campaigns, influencing social norms); SCT, which provided a structure for creating messages that model desirable behaviors and teach skills necessary to enact the behaviors (e.g., “Talk to your doctor about CRC screening”); and AAT, which suggested that messages should be proximal to opportunities to enact behavior for maximum impact (e.g., clinic-based reminders).

### 2.4. Media Campaign Intervention

The media campaign was conducted in the six intervention counties in Waves 2 and 4 of the study. The campaign in each county featured county-specific CRC survivors, individuals who had completed CRC screening, local physicians/nurses, and community members who were selected by the local community cancer coalition. The campaign images and messages were used in all campaign materials including billboard, posters, and articles sent to local newspapers. Although the billboard information was limited (slogan and photos of community members), the posters and newspaper articles included information about CRC, CRC risk factors and symptoms, CRC screening, and the message that CRC screening saves lives [15]. The billboard and posters were placed in high volume areas near the geographic center of each county, as determined by the local community cancer coalitions.

### 2.5. Clinic Intervention

Clinics within the six counties randomized to receive the intervention also received an intervention that included American Cancer Society (ACS) CRC educational posters and brochures in Wave 3 through the end of Wave 4 of the study. Clinic posters and brochures provided information about the mortality rates for CRC and motivational messages such as “If you're over 50, you need to get tested for colon cancer” and “Talk to your doctor about getting tested for colon cancer.” Local clinic managers were asked to display the ACS CRC materials in high visibility areas in waiting areas and exam rooms.

### 2.6. Comparison Group

The six comparison counties received a media campaign and patient education material in clinics related to healthy eating, “PEACHES” (Promoting Education in Appalachia on Cancer and Healthy Eating Styles), at the same time points the CRC screening intervention occurred in the intervention counties in Waves 2 through 4 of the study. The PEACHES campaign in each county featured local community members and farmers who were selected by the local community cancer coalition.

### 2.7. Study Timeline

The baseline participant recruitment began in September 2009 and was completed in April 2010. The media component of the intervention began in August 2010 and finished in July 2011. The clinic-based component of the intervention began in August 2011 and finished in July 2012. The combined intervention (i.e., media and clinic components) began in August 2012 and finished in July 2013. The final cross-sectional surveys (Wave 4) and final MRR were completed by December 2013.

### 2.8. Measures

The primary outcome was whether the participants were within the current U.S. Preventive Services Task Force (USPSTF) CRC screening guidelines for adults ages 50–75 (e.g., completed either an annual FOBT, a flexible sigmoidoscopy in the past five years combined with FOBT within the past three years, or a colonoscopy in the past 10 years) [10] as determined by MRR. The main independent variable was whether each participant lived in an intervention or comparison county.

### 2.9. Independent Variables

#### 2.9.1. Participant Demographic Characteristics

Participants provided information about their age, gender, race, ethnicity, marital status, education, household income, employment status, and health insurance.

#### 2.9.2. Participant Healthcare

Participants were asked about their comorbidities, CRC screening history, regular sources of medical care, and most recent CRC test (where the test and results were obtained).

#### 2.9.3. Perceived CRC Risk

To assess CRC risk, participants were asked “Compared to other men/women your age, what do you think your risk of getting colon cancer is in your lifetime?” Response was on a 5-point Likert scale (much lower, somewhat lower, about the same, somewhat higher, and much higher) [20]. Responses were dichotomized into high perceived risk (i.e., somewhat higher and much higher) and low perceived risk (i.e., much lower, somewhat lower, and about the same).

#### 2.9.4. Intention to Screen

Participants were asked (yes/no) if they were willing to have a CRC screening test if recommended by their doctor, have thought about talking to their doctor about completing a CRC screening test in the next year, intended to complete a CRC screening test in the next 6 months, and asked their doctor to order a CRC screening test.

#### 2.9.5. Participant-Reported Physician Actions regarding CRC and CRC Screening

Participants were asked (yes/no) if their doctor ever asked them about eating more fruits and vegetables, their family history of CRC, changes in bowel habits, rectal bleeding, and having a CRC screening test.

### 2.10. Process Evaluation

Process evaluation in Wave 2 involved a subset of participants (80 adults per county) responding to the mail-in survey asking if they had seen the campaign messages (billboards/posters used in the media campaign) during the past year. In order to ensure correct identification of campaign messages, pictures of fictitious CRC screening campaigns and similar questions addressing the sham campaign were included in the survey to serve as a control [15, 23]. Process evaluation in Wave 4 involved a subset of participants (80 adults per county) responding to a phone survey asking if they had seen the clinic-based educational materials (posters, brochures) during the past year.

### 2.11. Statistical Analyses

The primary outcome was being within guidelines for CRC screening at the end of each intervention period (as determined by MRR) and the time point of interest was Wave 4. Because 18% of the participants could not have their CRC screening status confirmed through a medical record, their screening status was imputed using a linear mixed model containing random county effects and fixed effects of predictors whose association with baseline screening status was significant at the 0.25 level or better as reported in Paskett et al. [16]. For each of the 50 imputed data sets, the proportion screened at Wave 1 and 4 was computed for each county. An ANCOVA model weighted by the inverse of the theoretical variance of the Wave 4 cluster means [24] was then used to compare Wave 4 screening rates between the intervention and comparison groups adjusting for Wave 1 screening rates and the results were combined across imputed data sets. As a sensitivity analysis, ANCOVA modeling was repeated for subjects whose medical record confirmed CRC screening status was observed (i.e., complete case analysis) and using self-reported CRC screening status. The same methods were used to compare intervention and comparison at Waves 2 and 3.

Linear models weighted by the number of participants in each arm at Wave 4 were used to explore the effect of the intervention on whether they talked with their doctor about family history of CRC, changes in bowel habits, rectal bleeding, and having a CRC screening test. The association between several patient/doctor interaction variables assessed at Wave 4 and CRC screening were assessed using multivariable logistic regression. Each behavior was included in a model that adjusted for county, marital status, insurance status, gender, smoking status, education, and employment. All analyses were performed using SAS v9.2 and v9.3 (SAS Institute, Cary, NC). Imputations were performed using the MMI_IMPUTE SAS macro [25].

## 3. Results

The demographic characteristics of participants (*n* = 4,491) by study wave in the intervention and comparison counties are presented in Table 1.

### 3.1. CRC Screening Rates

The estimated screening rates by wave are presented in Figure 2. The rates presented are averages across 50 imputed data sets. Participants from intervention counties were slightly more likely to have been within guidelines at Waves 1 and 4. However, after adjusting for baseline CRC screening rate, there was no difference in the Wave 4 screening rates between the intervention and comparison counties (*p* = 0.50). Wave 2 screening rates did not differ by treatment arm (*p* = 0.74), while participants in the intervention counties were less likely to be screened at Wave 3 than participants in the comparison counties (*p* = 0.02) controlling for the county-level rates in Wave 1.

### 3.2. Participant-Reported Physician Actions regarding CRC and CRC Screening

Of the 1,091 participants who completed the survey at Wave 4, 39 (6.9%) participants from the intervention counties and 40 (7.6%) participants from the comparison counties reported that their doctor asked them about their family history of CRC (*p* = 0.65). Fifty-six (9.9%) participants from intervention counties and 76 (14.5%) participants from comparison counties reported that their doctor asked about changes in their bowel habits (*p* = 0.009). A similar proportion of participants from intervention counties (8.1%) and comparison counties (9.0%) reported that they talked to their doctor about rectal bleeding (*p* = 0.64). One hundred ninety-two (33.9%) participants from intervention counties and 172 (32.8%) participants from comparison counties reported that they talked to their doctor about having a CRC screening test (*p* = 0.64). Lastly, a similar proportion of participants from intervention counties (85.1%) and comparison counties (81.9%) reported their willingness to have a CRC screening, if recommended by a doctor (*p* = 0.47, adjusting for baseline rate).

### 3.3. Predictors of CRC Screening

In separate multivariable models adjusting for county and demographic data (age, gender, race, ethnicity, marital status, education level, income, employment, and insurance), perceived CRC risk, intention to screen, and physician actions regarding CRC and CRC screening were statistically significant predictors of being within guidelines for CRC screening at Wave 4 (Table 2). Specifically, high perceived risk of CRC (OR = 1.79, 95% CI = 1.08, 2.95), willingness to have a CRC screening test if recommended by a doctor (OR = 6.23, 95% CI = 3.45, 11.27), and not thinking about talking to their doctor about a test in the next year (OR = 0.53, 95% CI = 0.35, 0.78) were associated with being within guidelines for CRC screening. Participants who asked their doctor for a CRC screening test (OR = 1.96, 95% CI = 1.13, 3.38) and talked to their doctor about eating more fruits and vegetables (OR = 1.47, 95% CI = 1.07, 2.03), family history of CRC (OR = 1.95, 95% CI = 1.11, 3.41), changes in bowel habits (OR = 1.86, 95% CI = 1.21, 2.87), and having a CRC screening test (OR = 1.82, 95% CI = 1.34, 2.46) were more likely to be within guidelines for CRC screening. Lastly, those participants whose doctors asked them to have a CRC screening test (OR = 10.02, 95% CI = 5.68, 17.69) were more likely to be within guidelines for CRC screening.

### 3.4. Process Evaluation

After the media campaign (Wave 2), 14.3% of the 502 participants from intervention counties reported seeing the correct billboard encouraging CRC screening. Of the 507 participants from intervention counties who answered questions about seeing the study posters, 12.4% reported seeing at least one of the three correct CRC screening posters. Odds of CRC screening were not greater among participants who reported having seen the correct billboard versus those who did not (OR = 0.87, 95% CI = 0.51–1.50), nor were they greater among participants who reported having seen at least one of the correct posters (OR = 1.42, 95% CI = 0.82–2.46, resp.), versus those who did not.

After the combined media and clinic campaign (Wave 4), 978 participants (503 intervention and 475 comparison) who reported having visited a doctor in the past year answered questions about seeing the clinic-based educational materials. Of the 503 participants from intervention counties who reported having visited a doctor in the past year, 57.9% reported seeing an ACS poster and 53.3% reported seeing a brochure about CRC screening at the doctor's office. There was no effect of reporting having seen either an ACS poster (OR = 1.34, 95% CI = 0.90–2.01) or a brochure (OR = 1.03, 95% CI = 0.69–1.52) on being within CRC screening guidelines.

## 4. Discussion

This group-randomized trial assessed the impact of a county-level intervention, consisting of media and clinic components, to increase CRC screening among Ohio Appalachian adults. The findings indicate that, despite a high willingness to have CRC screening, the intervention did not have an effect on CRC screening among the adults in the intervention counties, as approximately 35% of the participants had completed a CRC screening test in both the intervention and comparison counties. This result is similar to previously reported rates among Appalachian residents [15, 26–28]. Significant predictors of CRC screening within guidelines among participants were high perceived risk of CRC, willingness to have a CRC test if recommended by a doctor, doctor recommendation of a CRC screening test, and patient-physician communication about changes in bowel habits, family history of CRC, and eating fruits and vegetables.

We considered a number of possible explanations for the null results, including low exposure to the intervention. Participants may not have visited the locations where the posters and billboards were displayed. Process evaluation indicated that participants from the intervention counties were exposed to the clinic-directed intervention (i.e., 52% reported seeing the brochures); however, CRC screening rates did not differ between the two study groups suggesting that the media campaign and the clinic educational materials about CRC screening were not effective, as designed. Results of similar studies have raised questions about the efficacy of these types of interventions to bring sustained lifestyle changes and promote use of preventive health services [29–31]. When applied to a lower SES population with challenges related to health care access [9, 24, 28, 32], perhaps this media and clinic intervention only raised consciousness and intention (as demonstrated by previous media campaigns [11–13]) but could not lead to a major behavior change.

Future studies should consider utilizing media- and clinic-based interventions to increase knowledge and awareness of CRC screening coupled with personal contact from lay health advisors (LHAs) and patient navigators (PNs) to facilitate access to and completion of screening. LHA and PN interventions among underserved populations have been successful because they typically use trusted community members who understand the association between SES and cultural factors, as well as provider factors, associated with behavior change [33, 34]. With this knowledge, they serve as a bridge between the community and health care system by providing information, support, and encouragement [33, 34]. Previous studies using LHA and PN intervention programs to promote cancer screening have found significantly increased CRC screening rates [34–37]. Modeling these coordinated, targeted, and community-based programs in Ohio Appalachia could be similarly successful.

### 4.1. Limitations

The current study had several limitations. First, the overall rates of CRC screening in the clinics during the study were not measured. This would provide information about the potential for increasing rates of CRC screening among specific clinic patients. Also, we did not survey physicians about their recommendations for CRC screening and perceived barriers to CRC screening faced by their patients. This study utilized cross-sectional data which can limit the comparability across study waves and prohibits insight into the impact of the intervention. It is possible that people who completed the surveys after the clinic-based intervention (i.e., Wave 3) could have seen Wave 2 intervention material, causing a bias in their response. However, the main outcome was the comparison between Wave 4 and Wave 1 screening rates, and a cumulative effect of the interventions was expected. Lastly, study results may have limited generalizability because participants lived in one region of the US and were primarily non-Hispanic white.

## 5. Conclusion

This study tested the effectiveness of an intervention to increase rates of CRC screening among adults living in Ohio Appalachian counties. The county-level campaign consisted of media- (billboards, posters, and newspaper advertisements) and clinic-based (ACS brochures and posters) components about CRC and CRC screening. There were no differences in CRC screening rates between participants from the intervention and comparison counties at the end of the study, as measured by cross-sectional survey and MRR. Future research should examine how media- and clinic-based interventions can be modified to improve CRC screening rates among this underserved population.

## Figures and Tables

**Figure 1:** CONSORT diagram.

**Figure 2:** Unadjusted colorectal cancer (CRC) screening rates by intervention and comparison groups over time. Estimates are average over 50 imputed data sets.

**Table 1:** Participant characteristics by wave and study arm.

Variable	Level	Wave 1		Wave 2		Wave 3		Wave 4	
		Comparison (*n* = 562) *n* (%)	Intervention (*n* = 544) *n* (%)	Comparison (*n* = 601) *n* (%)	Intervention (*n* = 584) *n* (%)	Comparison (*n* = 547) *n* (%)	Intervention (*n* = 562) *n* (%)	Comparison (*n* = 525) *n* (%)	Intervention (*n* = 566) *n* (%)
Age	(mean ± SD)	61.7 (6.9)	61.2 (6.8)	61.7 (6.8)	61.7 (6.5)	61.4 (6.6)	61.6 (6.8)	62.4 (6.6)	62.6 (6.5)

Gender	Male	229 (40.7)	228 (41.9)	258 (42.9)	244 (41.8)	248 (45.3)	255 (45.4)	210 (40.0)	240 (42.4)
	Female	333 (59.3)	316 (58.1)	343 (57.1)	340 (58.2)	299 (54.7)	307 (54.6)	315 (60.0)	326 (57.6)

Race-White	No	20 (3.6)	15 (2.8)	21 (3.5)	17 (2.9)	28 (5.1)	23 (4.1)	31 (5.9)	21 (3.7)
	Yes	542 (96.4)	529 (97.2)	578 (96.5)	567 (97.1)	518 (94.9)	537 (95.9)	493 (94.1)	545 (96.3)

Hispanic ethnicity	No	553 (98.8)	541 (99.6)	591 (98.5)	575 (98.5)	546 (100.0)	555 (98.8)	515 (98.7)	562 (99.3)
	Yes	7 (1.3)	2 (0.4)	9 (1.5)	9 (1.5)	0 (0.0)	7 (1.2)	7 (1.3)	4 (0.7)

Marital status	Married	425 (75.6)	427 (78.6)	475 (79.0)	444 (76.0)	431 (78.9)	456 (81.1)	400 (76.2)	461 (81.6)
	Divorced/widowed	112 (19.9)	92 (16.9)	98 (16.3)	109 (18.7)	98 (17.9)	83 (14.8)	104 (19.8)	86 (15.2)
	Single	25 (4.4)	24 (4.4)	28 (4.7)	31 (5.3)	17 (3.1)	23 (4.1)	21 (4.0)	18 (3.2)

Education level	<High school	51 (9.1)	38 (7.0)	45 (7.5)	46 (7.9)	40 (7.3)	48 (8.5)	47 (9.0)	45 (8.0)
	High school	204 (36.3)	191 (35.2)	210 (34.9)	220 (37.7)	170 (31.1)	189 (33.6)	154 (29.3)	218 (38.5)
	Some college/college	307 (54.6)	313 (57.7)	346 (57.6)	318 (54.5)	336 (61.5)	325 (57.8)	324 (61.7)	303 (53.5)

Annual household income in last year	<$30K	163 (35.1)	144 (31.7)	150 (28.1)	188 (35.5)	159 (32.2)	159 (31.5)	168 (34.7)	187 (36.7)
	$30K–$60K	148 (31.8)	159 (35.0)	200 (37.5)	197 (37.2)	163 (33.0)	187 (37.0)	170 (35.1)	174 (34.1)
	$60K+	154 (33.1)	151 (33.3)	184 (34.5)	144 (27.2)	172 (34.8)	159 (31.5)	146 (30.2)	149 (29.2)

Employment status	Full/part time	252 (45.0)	239 (44.0)	270 (45.0)	250 (42.9)	237 (43.4)	248 (44.4)	205 (39.0)	231 (40.8)
	Retired/volunteer	219 (39.1)	209 (38.5)	222 (37.0)	239 (41.0)	222 (40.7)	227 (40.6)	234 (44.6)	254 (44.9)
	Disabled/unemployed	89 (15.9)	95 (17.5)	108 (18.0)	94 (16.1)	87 (15.9)	84 (15.0)	86 (16.4)	81 (14.3)

Insurance	Uninsured	49 (8.8)	48 (8.8)	61 (10.2)	62 (10.7)	40 (7.4)	54 (9.7)	51 (9.8)	46 (8.2)
	Public	217 (38.8)	192 (35.4)	220 (36.9)	222 (38.3)	186 (34.3)	206 (37.0)	226 (43.3)	248 (44.0)
	Private	294 (52.5)	303 (55.8)	316 (52.9)	296 (51.0)	316 (58.3)	297 (53.3)	245 (46.9)	269 (47.8)

**Table 2:** Multivariable logistic regression results for being within CRC screening guidelines (Wave 4)^a^.

Predictor	OR for CRC screening (95% CI)	*p* value
High perceived risk of CRC	1.79 (1.08, 2.95)	0.0233
Willingness to have a CRC screening test if recommended by doctor	6.23 (3.45, 11.27)	<0.0001
Thought about talking to doctor about completing a CRC screening test in the next year	0.53 (0.35, 0.78)	0.0016
Patient asked doctor for a CRC screening test	1.96 (1.13, 3.38)	0.0160
Talked to doctor about eating more fruits and vegetables	1.47 (1.07, 2.03)	0.0184
Talked to doctor about family history of CRC	1.95 (1.11, 3.41)	0.0199
Talked to doctor about changes in bowel habits	1.86 (1.21, 2.87)	0.0048
Talked to doctor about having a CRC screening test	1.82 (1.34, 2.46)	0.0001
Doctor asked patient to have a CRC screening test	10.02 (5.68, 17.69)	<0.0001

^a^Each variable was considered individually after adjusting for county and demographic factors. Each line represents a separate model. Results are from 30 multiply imputed datasets.
